The article "Awareness regarding Teledentistry among Dental Professionals in Malaysia" was published in 2022. Journal: Biomed Res Int.

# Awareness regarding Teledentistry among Dental Professionals in Malaysia

**DOI:** 10.1155/2022/3750556

**Published:** 2022-07-20

**Authors:** Romaisa A. Khokhar, Waleed A. Ismail, Adnan Sunny, Gul M. Shaikh, Sundas Ghous, Moeez Ansari, Syed Hamza Zia, Soban Arshad, Mohammad Khursheed Alam

**Affiliations:** ^1^Department of Oral Pathology, Shifa College of Dentistry, Shifa Tameer-e-Millat University, Islamabad 44000, Pakistan; ^2^Department of Periodontics, Shifa College of Dentistry, Shifa Tameer-e-Millat University, Islamabad 44000, Pakistan; ^3^Periodontics Unit, School of Dental Sciences, Health Campus, Universiti Sains Malaysia, 16150 Kubang Kerian, Kota Bharu, Kelantan, Malaysia; ^4^Department of Prosthodontics, Shifa College of Dentistry, Shifa Tameer-e-Millat University, Islamabad 44000, Pakistan; ^5^Department of Dental Education and Research, Shahida Islam Medical and Dental College, Lodhran 59320, Pakistan; ^6^Department of Dental Materials, Islamic International Dental College, Riphah International University, Islamabad 44000, Pakistan; ^7^Department of Periodontology, Rashid Latif Medical and Dental College, Lahore 54600, Pakistan; ^8^Department of Operative Dentistry and Endodontics, Foundation University College of Dentistry, Foundation University, Islamabad 44000, Pakistan; ^9^Orthodontics, Department of Preventive Dentistry, College of Dentistry, Jouf University, Sakaka, Al Jouf 72345, Saudi Arabia; ^10^Center for Transdisciplinary Research (CFTR), Saveetha Dental College, Saveetha Institute of Medical and Technical Sciences, Saveetha University, Chennai, India; ^11^Department of Public Health, Faculty of Allied Health Sciences, Daffodil International University, Dhaka, Bangladesh

## Abstract

**Objective:**

Teledentistry is considered to be a technological advancement in providing dental care to patients while effectively addressing the time management. Furthermore, the pandemic of COVID-19 has been here for quite long now, forcing the dental practitioners to ponder upon other methods of healthcare delivery apart from the traditional in-office direct clinical examination. The aim of this study was to explore the perceptions of dental professionals of Malaysia regarding teledentistry, which can act as a future pedestal for improvements in virtual dental practice and patient care.

**Materials and Methods:**

It was a descriptive, cross-sectional study involving an electronic survey of a sample of dental professionals of Malaysia. A prevalidated, 26-item, 5-point Likert-scale questionnaire was used in assessing the perceptions of dental professionals regarding teledentistry in four domains: existing concerns about teledentistry use, the potential of teledentistry in improving practice, usefulness of teledentistry for dental practice, and its usefulness for patients. Statistical analyses involved descriptive statistics which included frequency distributions.

The article "Awareness regarding Teledentistry among Dental Professionals in Malaysia" was published in 2022. Journal: Biomed Res Int.

**Results:**

An overall response rate of 31.0% was observed with 310 dental practitioners participating in the survey. More than 60% of respondents agreed that teledentistry would benefit the dental practice through enhancement of communication with peers, guidance, and new patients' referral. However, a substantial proportion of practitioners (70-80%) expressed uncertainty with accuracy of diagnosis, technical reliability, and privacy.

**Conclusion:**

Generally, the results of this study point towards the readiness of dental professionals of Malaysia to engage in teledentistry practice. However, further work needs to be done to assess the commercial feasibility of teledentistry, not only in Malaysia but also in other parts of the world. To start with, directed campaigns in reference to teledentistry are necessary to educate dentists and the public about the technology and its potential.

## 1. Introduction

In the last decade, tele-technology has picked up immensely in the medical and dental fields, providing a fast, safe, and more feasible way of delivering and sharing health information [1, 2]. Teledentistry specifically facilitates better referral systems based on consultation time, reduced waiting lists, decision-making, and patients' needs [3–5]. It can assist in extending dental care to the patients in rural areas while being more convenient and cost-effective, reducing the travel needs and ensuring proper referring channels [6]. Additionally, teledentistry can be of immense help in peer education, where clinical experiences can be shared among dentists, discussions and treatment planning sessions can be carried out, and continuous education sessions can be conducted through webinars and other online channels.

Despite telemedicine picking up pace in the field of healthcare and its use becoming very common, dental practitioners are still, unfortunately, not privy to the tremendous potential of teledentistry and how it can be adapted to cater to multiple sectors of dentistry. [7]. Past literature shows that several studies have been conducted to assess the perception of healthcare professionals regarding tele-health practices for the delivery of medical care to the patients. Palmer et al. assessed the perception of orthodontists on the implementation of digital technology, finding out that almost 70% of the respondents agreed with the use of tele-technology, and just about 36% had concerns with privacy and security issues [8]. In another study, Mandall et al. deduced that up to 71% of orthodontists agreed to the fact that teledentistry would be highly advantageous in patient referrals, and more than 50% of the respondents stated that teledentistry would help in considerable reduction of consultation timings [4]. Wood et al. conducted a study on the perception of general dentists and oral and maxillofacial surgeons towards teledentistry, where it was observed that a vast majority of participants agreed on teledentistry easing out patient access to healthcare, that too at a convenient cost [9]. In a study done to assess Australian dentists' perception towards teledentistry, Estai et al. concluded that almost 80% of the dentists agreed that the benefits derived from teledentistry's implementation are nothing but positive [10]. Patients' perception regarding teledentistry was also explored in a study, where Donelan et al. found out that a majority of patients (60%) reported no difference in the quality of consultancy provided through teledentistry, in comparison to the traditional in-person consultancy. It was also noted that most of the patients were of the opinion that teledentistry provides follow-up and care in a more convenient fashion [11].

The article "Awareness regarding Teledentistry among Dental Professionals in Malaysia" was published in 2022. Journal: Biomed Res Int.

In Malaysia, more studies have been published regarding telemedicine as compared to teledentistry. A study by Wan Maria Nabillah et al. evaluated the feasibility of teledentistry as a method for early detection of diseases. Their findings indicated that sensitivity and specificity of teledentistry in detecting lesions were high. Furthermore, it was observed that teledentistry was able to differentiate between malignant and nonmalignant lesions [12]. Another study by Oh et al. concluded that the there are multiple challenges faced by the induction of telemedicine in Malaysia, with most of the practitioners stating the cost, privacy concerns, and lack of technical training as the major areas of concern [13].

Surveys based on knowledge, attitude/awareness, and perception of respondents provide a greater understanding of the population towards the topic or problem at hand. These surveys are commonly used to identify knowledge gaps and behavioral patterns among sociodemographic subgroups to implement effective public health interventions [14]. These surveys can measure the extent of a known situation, confirm or disprove a hypothesis, and provide new tangents of a situation's reality. They can also establish the baseline for use in future assessments and help measure the effectiveness of health education activities' ability to change health-related behaviors. Apart from that, the perception studies can suggest an intervention strategy that reflects specific local circumstances and the cultural factors that influence them, which can assist to plan activities that are suited to the respective population involved [15].

The article "Awareness regarding Teledentistry among Dental Professionals in Malaysia" was published in 2022. Journal: Biomed Res Int.

Regarding Malaysian dental practitioners' perceptions and awareness towards teledentistry and its use in provision of healthcare, there is a dearth in past literature. Therefore, this was the primary aim of conducting this survey study, especially at a time when the COVID pandemic is forcing a work-from-home environment and use of technology is picking pace in almost every walk of life, especially in the field of medicine and dentistry.

## 2. Materials and Methods

### 2.1. Questionnaire Instrument

A prevalidated, electronic questionnaire was circulated among various dental practitioners of Malaysia between May and July of 2021. The questionnaire was adapted from a similar study by Al-Khalifa et al., which was conducted to assess Saudi Arabian dental practitioners' perceptions about teledentistry's usefulness and its role in improvement of dental practice and patient outcomes [16]. The first part of the questionnaire covered demographic information, as well as preferred methods of communication. The second part of the questionnaire was based on five-point Likert-type questions, with a total of 26 questions, further divided into four categories: practitioners' data security concerns, dental practice improvement through teledentistry, teledentistry being beneficial for dental practice, and its advantages for dental patients. Since this was a questionnaire-based study, an exemption was granted for this study by the ethical committee (JEPeM) of Universiti Sains Malaysia, Health Campus, Kelantan, Malaysia.

### 2.2. Questionnaire Distribution

This was a cross-sectional survey study. An e-mail list of 1000 random dental professionals was obtained from the Malaysian Dental Council (MDC) database, on the condition of keeping all the data confidential and maintaining anonymity. The MDC database contains information of almost 12,000 dental professionals of Malaysia. It was ensured that this random sample was synonymous to the general Malaysian dental workforce in demographic as well as professional features. Furthermore, stratification of the sample was done based on gender and qualifications, in order to attain a true sample of the Malaysian dental practitioners. The survey questionnaire was then distributed to the sample participants via e-mail. The questionnaire comprised of definition of teledentistry and briefly explained the study's purpose. This was succeeded with an informed consent form prior to participation in this survey, which was solely on volunteer basis. An e-mail of reminder was set to be sent on weekly basis to the nonresponding members.

The article "Awareness regarding Teledentistry among Dental Professionals in Malaysia" was published in 2022. Journal: Biomed Res Int.

### 2.3. Data Analysis

The data were entered in MS Excel by Office 365 (Microsoft Corp., USA) and transferred to IBM SPSS Statistics for Mac version 26 (IBM Corp., Armonk, NY, USA) for statistical analysis. Descriptive statistics included frequency distributions.

## 3. Results

Between May and July 2021, survey questionnaires were e-mailed to 1000 random Malaysian dental practitioners. A total of 310 e-mail replies were received, indicating a response rate of 31.0%.

### 3.1. Demographic Characteristics of Respondents

Nearly 60% of the respondents were in the age range of 25 to 34 years. Almost half of the respondents were general dental practitioners, more than 60% being males, and two-thirds of them had less than five years of work experience. Majority of the practitioners worked in major cities (64.5%), and the remainder were working in smaller cities and towns of Malaysia. Almost one-third of the respondents (32.3%) worked 1–19 hours per week. More participants were working in private practices (35.5%), which was followed by those working in both (public and private) practices concomitantly (25.8%), and then, came those working at solely academic practices (22.6%) (Table 1).

### 3.2. Preferred Methods of Communication

There has been drastic alteration in the modes of preferred communication with the advent of tele-technology, as traditional methods of communication, including facsimile or letters, seem to be very less or nonpreferable now. The most popular methods of communication chosen by the participants were as follows: in-person contact (48%), telephone (29%), social media (16%), and e-mail (6.5%). The least chosen (or almost nonpreferred) modes of communication among the practitioners were the usage of letters or facsimile and videoconferencing.  Figure 1 depicts how the respondents chose their preferred methods of communication. As there was no compulsion on choosing multiple options, therefore, it was best to present the data in the form of a bar chart.

### 3.3. Teledentistry Confidentiality and Security Issues

When data are sent online, potential forgery of the digital data becomes a larger cause of concern than patient confidentiality, obtaining patient consent, software and hardware incompatibility, or reliability of equipment. This was evident from the results of this study as well where over 90% of respondents showed concern regarding digital forgery. This was followed by concerns with patient confidentiality, where about 84% of respondents expressed significant concerns. After this were the concerns regarding incompatible software and hardware and on reliability of tele-dental equipment, where almost 80% of respondents expressed significant concerns. The comparatively lowest levels of concern were seen in respect of gaining patient consent for teleconsultation, with a little over 70% of participants showing concern towards gaining patient consent (Table 2).

The article "Awareness regarding Teledentistry among Dental Professionals in Malaysia" was published in 2022. Journal: Biomed Res Int.

### 3.4. Teledentistry and Practice Improvement

Most of the respondents were of the opinion that teledentistry would improve dental practice in multiple aspects. More than 70% of respondents were in agreement that teledentistry will assist in more efficient referrals, will shorten the waiting lists at dental practices, and will provide a safer working environment for dentists, a notion of particular importance during the pandemic. A clear majority (58%) agreed that teledentistry would assist in improving interaction between colleagues as well. However, on the flip side, 42% of the participants felt unsure about the diagnosis' accuracy using teledentistry in a clinical setup (Table 3).

### 3.5. Teledentistry Usefulness for Dental Practice

In accordance with majority of participants, it was deduced that teledentistry would be beneficial to a dental practice by enhancing continuing education and clinical training and would be more timesaving in comparison to a conventional referral system. Almost 42% of the respondents felt that the costs of dental practice would be reduced considerably with the implementation of teledentistry, but extratime would be required in arranging special appointments for dental photographs. On the contrary, almost half of the participants were very less or not convinced upon teledentistry increasing treatment time spent with the patient. There was a mixed opinion on whether setting up infrastructure for teledentistry would be too costly (Table 3).

### 3.6. Teledentistry Usefulness for Dental Patients

There was a unanimous agreement by majority of dental practitioners (60%) over teledentistry being beneficial to the patients. In support of this, almost 75% of respondents were of the opinion that teledentistry would specially be advantageous for patients residing in remote or rural locations. The same proportion of practitioners also agreed on few other patient benefits from teledentistry, including patient education and reduction in the dental clinic visits, and they opined that health insurance plans should have a covering for teledentistry. The rest of the questions aimed at assessing benefits of teledentistry for patients showed a fairly positive response, where over 54% of participants agreed that teledentistry would improve communication with patients, would be beneficial in monitoring the patient's condition, and would be convenient and well received by patients. However, almost half of the practitioners were unsure whether teledentistry would save money for the patients (Table 3).

The article "Awareness regarding Teledentistry among Dental Professionals in Malaysia" was published in 2022. Journal: Biomed Res Int.

The final question of this survey addressed the dental specialties where practitioners thought teledentistry would be most well suited. Community dentistry and dental hygiene came first, with over 70% of the response. This was succeeded by oral medicine (58%), pedodontics (48%), and oral radiology (40%). The remaining dental specialties got lesser than 40% of the response from the participants (Figure 2).

## 4. Discussion

This study is probably the first of its nature to investigate Malaysian dental practitioners' perceptions of teledentistry's usefulness in different practical aspects of dentistry. Overall, a good proportion of dental practitioners unanimously agreed on tele-technology being beneficial for dentistry. Most of the practitioners (70%) believed that teledentistry would be advantageous to patients (especially those residing in remote locations), most importantly by avoiding unnecessary visits to the dental practice. They also agreed on the fact that teledentistry would be of great assistance in patient education. Generally, the results of this study are in support of the benefits teledentistry has for both the patients and the dental practice. Other published studies based on perceptions of dental practitioners about teledentistry have deduced the same results, where majority of respondents agreed on the benefits of teledentistry, especially for the patients and the dental practice [10, 17]. Though the difference in our study compared to previous ones is very slight, it might be related to the study participants' other concerns regarding the advantages to the patients.

Similar to some previous studies, there was considerable doubt regarding teledentistry being able to provide accurate diagnosis as compared to in-person consultancy [4, 5, 18–20]. Some of the studies though depicted a high level of diagnostic accuracy with oral pathologies or dental caries [18, 21]. This was a result of proper training; the sessions were conducted by practitioners for proper diagnosis. Therefore, it is possible for teledentistry to produce an acceptable diagnosis, given that adequate training following a set protocol is administered. Almost 65% of the respondents indicated that for photography in teledentistry, an additional visit would be necessary. This depicts the practitioners' need for trained personnel in order to take proper photographs [10]. This requirement can also be minimized if proper dental photography training sessions are undertaken by the practitioners. The highest reported concern (90%) was regarding potential digital forgery. Sharing health information over the Internet is always a matter of concern for patients as well as for practitioners, as to who can view or access the information, and this comes in agreement with few past studies [19, 22, 23]. However, the majority of participants agreed upon the fact that teledentistry will help in reduction of waiting lists, a benefit which can be attributed to effective referral process through teledentistry. Another important advantage of teledentistry which got highlighted was improvement in guidelines and peer communication. This means that the patients will ideally be referred to a specialty clinic based on an informed decision, keeping in mind each patient's condition and needs. For this reason, patients' referral process and management are two of the integral driving forces in implementation of tele-technology in dental practice [24–27].

The article "Awareness regarding Teledentistry among Dental Professionals in Malaysia" was published in 2022. Journal: Biomed Res Int.

Respondents were generally unanimous about the advantages to the dental practice as a result of teledentistry implementation. They opined that foremost, it would be beneficial in education and professional training of dental staff for practices. The dental personnel, through distance learning, could benefit from targeted information whenever required, thus having an improvement in their knowledge and skills [28–30]. The respondents also agreed that teledentistry would be timesaving and reduce overhead costs at a dental practice. Efficient time management and reduced costs can attract patients and gain their trust. Multiple past literatures deduced that teleconsultations bore a low cost in comparison to traditional face-to-face consultations [19, 31, 32]. The majority of the respondents (70%) agreed that teledentistry should be inculcated into health insurance plans, which can act as an incentive to attract patients. Many countries have already included telepractice and teleconsultation into different dental insurance plans [33–35].

Participants showed high concerns relating to digital forgery (90%), digital security (85%), hardware being incompatible, and reliability of the equipment (80%). Having the latest digital technologies is of no use without the proper infrastructure design. For its resolution, compatible hardware and software need to be implemented in order to ensure entirely secure integration between technical components. An appropriate infrastructure and setup will not only prevent/minimize the technical errors in digital operations but will also help in cutting down costs effectively [8, 34–37].

When inquired about the dental specialties which can benefit the most from teledentistry, the majority of the respondents selected community dentistry and dental hygiene, followed by oral medicine and pedodontics, and just over 40% of the participants selected oral radiology. This goes on to signify a rather single-track vision of the practitioners, where the general perception about teledentistry's implementation is limited to screening, diagnosis, or patient education. Recent advancements have proven though that if used appropriately, teledentistry holds the potential for successful treatment, postoperative care, and effective treatment planning as well. Thus, directed campaigns regarding teledentistry are needed to widen the perception of practitioners, explaining the full spectrum of teledentistry and its applications.

The article "Awareness regarding Teledentistry among Dental Professionals in Malaysia" was published in 2022. Journal: Biomed Res Int.

Starting from the year 2021, most of the dental practitioners shifted their practice to teledentistry, based upon teleeducation and teleconsultation, essentially to cope with the COVID-19 pandemic [38, 39]. To gain control over its spread, routine dental care has majorly been canceled during the pandemic, either by the respective governing medical/dental bodies or by practitioners themselves [40–42]. In such circumstances, an excellent pedestal is set for the use and progression of teledentistry in dental practices to ensure continuity of adequate dental care to the patients, keeping in check the safety against the pandemic simultaneously.

Relatively higher number of questions in the questionnaire can be thought of as a limitation of this study. A more precise questionnaire might even show better response rate. The relatively low response rate can also be accounted for the fact that the data for this study was completed in 2 months time (May to July 2021) as the pandemic was at its peak then. Another limitation can be the use of 5-point Likert scale, as multiple studies have reported psychologic barriers that respondents tend to choose the middle value as a safe, moderate choice rather than opting any value on either of the extremes. This might affect the actual awareness and perception levels of the respondents [43, 44].

The results of this study show positive perception and attitude of Malaysian dental professionals towards teledentistry as a general concept. However, further studies need to be conducted based on efficacy of patient screening, diagnosis, and referral by the use of teledentistry. Similarly, a study on the readiness and willingness of Malaysian dental patients towards teledentistry needs to be done in order to assess the feasibility of its implementation.

## 5. Conclusion

Generally, the feedback from this survey depicts readiness of the dental practitioners of Malaysia to implement teledentistry commercially in dental practices. Despite showing few concerns, the majority of the respondents agreed with the general concept and displayed a high understanding of the ethical and technical limitations while using teledentistry. However, further investigation is needed for understanding potential challenges dental practices and institutes can face during teledentistry implementation, so as to try and overcome them. Also, professional training regarding the implementation of teledentistry needs to be commercialized and made widespread.

The article "Awareness regarding Teledentistry among Dental Professionals in Malaysia" was published in 2022. Journal: Biomed Res Int.

## Figures and Tables

**Figure 1:** Preferred communication tools among dental practitioners.

**Figure 2:** Preferred dental specialty for application of teledentistry.

**Table 1:** Demographic and professional characteristics of respondents.

Sample characteristics	Frequency	%
Age (in years)		
25-34	186	60.0
35-44	48	15.5
45-54	42	13.5
55-64	31	10.0
>65	3	1.0
Gender		
Male	190	61.3
Female	120	38.7
Qualification		
Specialist	70	22.6
General dental practitioner	140	45.2
Resident/graduate	100	32.3
Dental therapist	0	0.0
Work experience (in years)		
0-5	196	63.2
6-10	79	25.5
11-15	29	9.4
>16	6	1.9
Location of the main job		
Major city	200	64.5
City/town	90	29.0
Remote area	20	6.5
Work setting of the main job		
Private	110	35.5
Public	50	16.1
Both (private and public)	80	25.8
Academic	70	22.6
Working hours (per week)		
1-19 hours	100	32.3
20-34 hours	60	19.4
35-49 hours	90	29.0
50-64 hours	30	9.7
>65 hours	30	9.7

**Table 2:** Concern of practitioners regarding data security and patient consent.

Questions	VC (%)	LC (%)	NA (%)	NP (%)	NC (%)
Gaining patient consent for teleconsultation	48	23	16	10	3
Confidentiality when data are sent online	61	23	7	6	3
Potential for digital forgery	61	29	7	—	3
Incompatible hardware and software	39	42	6	13	—
Reliability of teledental equipment	42	39	19	—	—

VC = very concerned; LC = little concerned; NA = not feeling either way; NP = not particularly concerned; NC = not concerned at all.

**Table 3:** Practitioners' perceptions of benefits of teledentistry in improving dental practice and patient care.

Questions	SD (%)	D (%)	N (%)	A (%)	SA (%)
*Practitioners' perception of the capability of the teledentistry to improve practice*					
Teledentistry would provide accurate diagnosis in a clinical setting	10	16	42	32	—
Teledentistry would help shorten the waiting list	10	10	3	71	6
Teledentistry would enhance guidelines and advice	10	10	13	61	6
Teledentistry would improve the interaction between peers	10	16	16	58	—
Teledentistry would provide a safe atmosphere for practicing dentistry	10	3	3	48	36
Teledentistry would make patient's referral more efficient	9	10	13	55	13
*Practitioners' perception of the usefulness of the teledentistry for dental practice*					
Teledentistry would enhance clinical training and continuing education	13	9	26	52	—
Teledentistry would reduce costs for the dental practices	10	13	35	36	6
Teledentistry would increase treatment time spent with the patient	10	23	19	42	6
Teledentistry would necessitate an extra appointment for taking photographs	—	19	16	49	16
Teledentistry would save time compared with a referral letter	—	—	42	48	10
Teledentistry would be too expensive to set up	—	32	36	32	—
Teledentistry would provide adequate diagnostic information	—	26	13	58	3
*Practitioners' perception of the usefulness of the teledentistry for patients*					
Teledentistry would save money for patients	—	16	42	36	6
Teledentistry would improve communication with patients	—	29	16	55	—
Te5ledentistry would be helpful in patient education	—	—	23	68	9
Teledentistry would help to avoid unnecessary travel to dental clinic	—	—	13	58	29
Teledentistry would be helpful in monitoring the patient's condition	—	13	29	55	3
Teledentistry would be convenient and well received by patients	—	—	39	61	—
Teledentistry would be useful for patients in remote areas	—	7	19	58	16
Teledentistry should be covered by dental insurance plans	—	3	26	55	16

SD = strongly disagree; D = disagree; N = neutral; A = agree; SA = strongly agree.

The article "Awareness regarding Teledentistry among Dental Professionals in Malaysia" was published in 2022. Journal: Biomed Res Int.

## Data Availability

The data that support the findings of this study are present in the manuscript.
